RETRACTED

# Research on the Influence of DNN-Based Cross-Media Data Analysis on College Students' New Media Literacy

**DOI:** 10.1155/2022/9224834

**Published:** 2022-08-03

**Authors:** Rui Xu, Chen Wang, Yen Hsu, Xinyan Wang

**Affiliations:** ^1^The Graduate Institute of Design Science, Tatung University, Taipei, Taiwan 11604, China; ^2^School of Art and Design, Fuzhou University of International Studies and Trade, Fuzhou, Fujian 350200, China; ^3^College of Journalism and Communications, Shih Hsin University, Taipei, Taiwan 11604, China; ^4^Nanhang Jincheng College, Independent College of Nanjing University of Aeronautics and Astronautics, Jiangning, Nanjing 211156, China

## Abstract

New media has gradually become the mainstream media that college students rely on, and new media has also brought about subversive changes and has become an essential medium for college students to receive and disseminate information, such as learning, interpersonal communication, and entertainment. Young college students have become the most enthusiastic recipients and users of new media. College students need to have the ability to recognize, understand, and criticize new media. New media literacy has become the basic quality that every college student living in modern society must have. This paper takes 826 college students as the research object with deep neural network (DNN), and then analyzes their media selection tendency, media usage time, positive influence, and the relationship with new media literacy. The formation of good new media literacy has a positive effect and influence on the work and study after the university, making it the main force of the media society.

## 1. New Media

The media is the medium of dissemination of information [1–3]. It refers to the tools, channels, carriers, intermediaries, or technical means that people use to transmit and obtain information, as well as the tools and means to transmit text, voice, and other information. The media can also be regarded as all technical means to realize the transmission of information from the information source to the recipients. The traditional four media are televisions, radios, newspapers, and magazines.

With the development of the Internet, new media has been updated and upgraded. So far, considering different research perspectives and levels, the definition of new media in academia has not been unified. New media is a relative concept. New media can be regarded as the product of new technologies. The latest technologies such as digitalization, multimedia, and network are all necessary conditions for the emergence of new media. After the birth of new media, the form of media communication has undergone earth-shaking changes, such as subway reading, large screens in office buildings, and so on, all of which have transplanted the communication content of traditional media into a new communication space.

RETRACTED

New media can be divided into four types [4, 5]: mobile media, digital TV, online new media, and outdoor new media. The new media represented by mobile smart phones is the new media with the largest user scale and the most convenient use. Smartphones help people download and install the APP they need by connecting their smart phone to mobile data at any time and place. You can freely choose the APPs and applications you need on your smart phone, and people's needs for office, life, leisure and entertainment, payment, communication, and so on, can be met on the mobile smart phone client. Digital TV is developed based on Internet technology, including new media forms such as digital TV and Internet Protocol TV. People can enjoy more resources and services through digital TV media. New online media include online TV, blogs, podcasts, videos, e-magazines, and so on. Outdoor new media uses LCD TV as the carrier, such as bus TV, subway TV, aviation TV, large LED screen, and so on.

### 1.1. New Media Literacy

Media literacy [6] is the ability to receive, understand, integrate, judge, analyze, and evaluate information disseminated by traditional media such as television, magazines, radio, and newspapers. In the age of traditional media, people play more of the role of information consumers for oral communication, written expression, and image information. The boundary between information producers and information consumers is clear, there are few ways for individuals to participate in information production, and information dissemination is only a one-way dissemination. Therefore, traditional media literacy is proposed for the role of individuals as consumers of information.

New media literacy is divided into functional access and critical access [7]. Each dimension is refined into specific capabilities, and functional access includes access skills and understanding, mainly the ability to acquire, accept, and understand information. Critical access includes analysis, integration, and evaluation, emphasizing the ability to criticize and question media information. Functional creative use includes creative skills and production, that is, you can master the technology of creating media content, use the media to disseminate information, and communicate and share your insights with others. Critical creativity includes participation and creation, emphasizing participation in social interaction and the ability to think rationally and critically to create meaningful media content.

RETRACTED

With the continuous development of new media technology, new media is no longer concentrated in a few elite groups, and the general public has become the main user group of new media, which has also brought earth-shaking changes to the media industry. At this time, individuals play the roles of information transmitters and producers, and the connotation of new media literacy should be further enriched and improved.

When people use new media correctly and efficiently, new media can better serve people's work and life. With new media to actively participate in social interaction, constantly improve yourself in social interaction, and gradually enhance the awareness of concentric circles, responsibility awareness, civilized online awareness, and network security awareness. In general, new media literacy mainly includes the ability to acquire and understand, to think and question, to participate and create, and to use and produce.

### 1.2. MOOC Course—*New Media Literacy*

In China's university education system, *Sun Yat-sen University* first opened a new media literacy course for college students on the MOOC platform in 2014. The course has successfully completed 12 rounds, each of which is divided into 9-week lesson plans, focusing on the Internet revolution and its impact, future journalism and future audiences, and online public opinion. The course outline displayed on the official MOOC [8] platform is shown in Table 1.

The course *New Media Literacy* is taught by MOOC as an official platform, and the main body is students from various universities in China. At the beginning of each semester, college students can freely choose whether to participate in this course or not. Many students in the course said that the course attaches importance to multiple perspectives and broad vision and focuses on the introduction and discussion of fresh cases. They know how to use the Internet more rationally and maturely. Many noncollege students also agree with this view, saying that the course has helped them build the necessary network literacy.

## 2. Analysis and Retrieval of Cross-Media Data

The technology of cross-media data processing [9] focuses on intelligent information retrieval, analysis and reasoning, knowledge graph construction, and intelligent storage and applied to cross-media intelligent publication publishing, intelligent management of archives information, smart city construction, education trend forecasting, and so on. China attaches great importance to the deep integration of intelligent technology and education and continues to promote the exploration and innovation of intelligent technology in education. By developing key technologies, constructing application models, summarizing practical cases, and integrating cross-media information retrieval, knowledge graph construction, and intelligent storage, the application of cross-media intelligent technology in the field of education is deepened.

RETRACTED

### 2.1. Cross-Media Topic Detection

In the past 10 years, people from all walks of life have invested a lot of human resources and financial support for the processing of massive text, image, and video cross-text data. However, without effective abstraction techniques, it is difficult for users to digest the hot topics and key information they care about. Integrating cross-media information [10] into topics provides users with an easy way to understand real events that have occurred and enhance user experience. Cross-media topic detection is a technique for summarizing unstructured cross-media data. Text topic detection has been unable to meet the needs of users to vividly browse hot topics and understand the growing network of multimedia data. Cross-media topic detection has become the focus of research.

Topic model is a generative model based on probability graph, which is widely used in topic detection tasks by establishing the association between information and topics.

Latent Dirichlet Allocation [11] was first proposed in 2003. The LDA model is suitable for *latent semantic analysis* of data and is widely used to identify hidden topic information in large-scale corpora, giving each document in the corpus. LDA does not require prior knowledge between documents and topics nor does it require a trained corpus. Topic model-based cross-media topic detection mostly improves the classic LDA model. LDA believes that there are several topics in a document, and each topic corresponds to different words with different probability distributions. For the generation process of a document, first select a topic from the probability distribution of a document topic and then select a word under the selected topic with a certain topic word probability distribution as the generated the first word in the document. Then repeat the word generation process to generate a complete document.

Cai et al. [12] studied multimodal topic detection on Twitter, using various visual features to study the impact of Twitter images on social topic detection for different topic categories. A space–time multimodal Twitter LDA topic model is proposed to extract five different Twitter features, including text, images, timestamps, locations, and hashtags, from raw tweet streams and feed them into the STM-Twitter LDA model, aiming to discover lots of tweets on the topic.

Klan proposed an automatic summarization framework [13] for multimedia social events to automatically generate visual summaries in microblog streams of multiple media types. First, the noisy data are removed, and an efficient spectral filtering model is used to estimate the relative probability of an image to a given event, and a noise removal method is designed to remove images that may be noisy.

RETRACTED

Wang et al. [14] proposed Image-regulated Graph Topic Mode, the main idea is to use the corresponding image to model text into the semantic space through latent features. IGTM is a generative probabilistic model that combines weakly supervised information based on weighted image graphs. By building weighted image graphs, IGTM can discover explicit text–image relationships and latent text–image relationships to discover potential topics.

### 2.2. Analysis of Transmedia Perspectives

Opinion analysis [15] is also known as opinion mining; its main goal is to identify the user's opinion categories and sentimental tendencies, which correspond to the research of opinion clustering and the research of sentiment analysis, respectively. In cross-media public opinion analysis, opinion clustering is generally aimed at textual modalities, which is to classify and summarize comments made by users on the Internet about certain topics or policies.

For topic text clustering, the text clustering of college students' media topics is to group similar topic documents into one category, and the similarity of documents in different categories is low. Generally, the topics of college students are not known in advance, so clustering algorithms are mostly used. Text clustering can be divided into three stages: text preprocessing, feature representation, and clustering. In the preprocessing stage, unstructured text data are converted into computer-processable structured data, generally including removal of stop words, punctuation, and word segmentation, among which word segmentation is to process Chinese text. In specific operations, corresponding methods are adopted according to different tasks. In the feature representation stage, the preprocessed structured data are represented in a specific form for computer processing, which generally includes feature dimension reduction, feature space establishment, and weight representation. In the final cluster analysis stage, according to the similarity between documents, clustering is performed according to certain rules. The commonly used clustering algorithm is k-means. The general process of college students' cross-media topic text clustering is shown in Figure 1.

Sentiment analysis [16] is divided into text sentiment analysis and visual sentiment analysis. There are three sentiments, such as positive, negative, and neutral. Multicategory topic sentiment categories include anger, disgust, fear, surprise, happiness, sadness, and neutrality. The main task of text sentiment analysis is to identify which emotions are carried by college students' media speech. Among them, the main work of visual emotion analysis research is to identify emotions based on facial expressions of people in pictures or videos.

RETRACTED

Among the common methods of text sentiment analysis, machine learning and dictionary-based methods are the main ones. When applying machine learning methods to college students' cross-media sentiment analysis, supervised learning methods, namely classification algorithms, are used. The classification algorithm contains two sets of documents of training set and test set. The classifier uses the training set to train various parameters of the model and then uses the trained model to verify it on the test set. For example, decision tree algorithm and support vector machine algorithm are used for sentiment analysis of college students.

### 2.3. Deep Neural Network

In recent years, deep neural network (DNN) has been favored by researchers in cross-media retrieval. The Deep Restricted Boltzmann Machine [17] models joint representations across different modalities by learning spatial probability densities over multimodal inputs. Deep Canonical Correlation Analysis aims to find suitable nonlinear transformations to make the underlying features highly linearly correlated between different modal data. Inspired by the efficiency of convolutional neural networks in image and text processing, some scholars proposed the Deep and Bidirectional Representation Learning Model [18], which uses two different types of convolutional neural networks to represent text and image. DNN and its improved models have demonstrated excellent performance in multiple cross-media detection tasks. Cross-media data retrieval and analysis with deep neural network as the main technology has also been well applied and promoted in college students' new media literacy.

An important characteristic of deep neural network is that its “depth” is larger than the general neural network model, and it is composed of “input layer, hidden layer, and output layer.” Deep neural networks mainly include deep trusted networks, constrained Boltzmann machines, convolutional neural networks, and so on. In this paper, convolutional neural network is studied, and on this basis, its related parameters are modified; a new DNN is constructed, and DNN is used for the identification of traffic signs, so as to study the influence of different network structures on its performance.

The convolutional neural network is a type of neuron that researchers have discovered by observing the cerebral cortex of cats that can reduce the complexity of the feedback neural network. CNN technology is widely used in pattern classification because it does not need explicit feature extraction of images and can directly train the original images.

RETRACTED

The network of DNN is generated by multiple convolutional layers and a sample layer alternately, and each neuron is only connected to the neuron of the previous layer. It is a multilevel feature extraction method. It inputs the initial pixel intensity of the image into DNN, obtains feature vectors through feature extraction of convolution layer and subsampling layer, and then classifies them through fully connected output neurons.

Compared with the conventional neural network structure, DNN has more hidden layers [19], as shown in Figure 2. Inside the DNN, the input layer receives various media data collected, and the middle layer processes the text or image media data and outputs it from the last layer. Except for the first and last layers, the middle layers are hidden layers. The *n*_th_ layer and the (*n*+1)_th_ layer are fully connected, that is, any two neurons are connected.

From a local point of view, it can be understood as a combination of multiple linear relationships and activation functions. Taking the Sigmoid activation function as an example, the relationship is as follows.

(1) $$\begin{array}{c} \left\{\begin{array}{c} f\left(x\right)=w_{i}x_{i}+b,\\ f\left(z\right)=\frac{1}{1+e^{-z}}. \end{array}\right. \end{array}$$

## 3. Cross-Media Data Analysis of College Students Based on DNN

According to China's New Media Development Report 2020-2021 [20], the digital economy has become an important driving force for building a new development pattern, Internet governance has strengthened special rectification and platform management, and the construction of digital China has been promoted with high standards and high quality. The development trend of new media in China as shown in Figure 3.

### 3.1. DNN Optimization Design

In the experiment of this paper, each DNN is modified accordingly, and a plurality of DNNS is constructed according to the results of the experiment, and a plurality of DNN fuzzy discriminant matrices is constructed according to the results of the experiment, and the output of each data set is comprehensively judged according to the principle of fuzzy mathematics, so as to determine the final category.

#### 3.1.1. Modify the Size of the Convolution Kernel

The convolution kernel slides on the input image, and the center of the convolution kernel is always consistent with the pixels of the image. During sliding, the convolution kernel will perform operations with all pixels of the image and finally take its corresponding position as the output. On this basis, small feature images can be obtained by using rolling Windows for superposition. On this basis, the convolution kernel size of the convolution layer is adjusted sequentially, and a large number of experimental data are compared to obtain the best network architecture.

RETRACTED

#### 3.1.2. Modify the Size of the Subsampling Window

Subsampling is mainly through the subsequent specialization of the features obtained by convolution, so that the features input a small number of features into the convolution layer, so that the size of the sample window has a great influence on the recognition effect of neural network. The general size of the subsampling window is 2 × 2. Therefore, without overlap, the size of the subsampling window can be adjusted by the characteristic curve of the convolution layer.

#### 3.1.3. Modify the Number of Batch Samples

Batch sampling number refers to the training samples that are divided into several groups; each group is trained separately, distributed on the network, and then the weight is updated, so that all the training samples will be included in each learning cycle. In a large number of sample data, the selection of appropriate batch sample number will have a great impact on the weight of neural network and the effectiveness of network recognition.

#### 3.1.4. Modify the Number of Feature Maps

The number of feature graphs represents the number of convolutional kernels used by the convolutional layer and the feature types extracted from the convolutional layer. Therefore, the number of feature graphs of the convolutional layer plays an important role in subsequent recognition. In order to test whether the change of the number of feature maps has any influence on the recognition effect of neural network, the experimental data are used to test the change of feature maps. The number of feature graphs in the first convolution *C*1 is taken as a constant value and changed in the second convolution *C*2, so as to obtain the best experimental results.

#### 3.1.5. Fuzzy Decision Output

The concept of fuzzy mathematics is subordinate to nonabsolute, while the output of DNN is fuzzy. Therefore, the output of MCDNN is evaluated comprehensively by fuzzy mathematics.

The pseudocode of this optimization model is as follows in Algorithm 1.

### 3.2. Media Choices Preferred by College Students

Taking 826 college students as the research object, among the three most favored media, the Internet accounts for the highest proportion, followed by television, and finally newspapers and periodicals. The three types of media selected accounted for 73%, 59%, and 31%, respectively. The new media represented by network media is an indispensable and most in-demand type of media in the life of college students, and its important role is self-evident. Three media commonly used by college students as shown in Figure 4.

RETRACTED

The distribution of Internet media usage time among students: the proportion of college students who spend 11–20 hours online per week is 37%, the proportion of 21–30 hours is 25%, and the total proportion of more than 30 hours or less than 10 hours is 38%. Wechat, Weibo, forums, and games have become the main channels for students to obtain online information. The weekly media time of college students is as shown in Figure 5.

### 3.3. The Positive Impact of New Media on College Students

New media provides a platform for college students to express themselves and express their hearts [21, 22]. College students who grew up in the information age generally have independent and assertive personalities. They have a high demand for the timeliness of information transmission and feedback in communication, the breadth, and freedom of communication. New media provides a convenient communication channel for college students. At the same time, it greatly broadens the channels for college students to acquire knowledge. For example, a large amount of information is obtained through electronic magazines, official platforms, social accounts, and so on, which invisibly enhances the self-learning awareness of college students and obtains useful information for themselves. The new media expands the interpersonal circle of college students, enriches the daily behavior of college students, and conveys information quickly and effectively through audio and video files.

### 3.4. The Relation between Transmedia Use and College Students' New Media Literacy

Among the surveyed college students, according to their concerns about the topics, current affairs hotspots and processing methods in the use of cross-media [23]. Under the background of DNN, the new media literacy, interpretation ability, critical questioning ability, independent thinking ability, and verification reporting ability of college students are analyzed from these aspects.

#### 3.4.1. In-Depth Interpretation

About one-third of college students are slightly lacking in their ability to understand and process information. When faced with the wave of new media information, it is easy to follow the public to receive or receive information in a comprehensive manner. Even many college students spread unverified information on various media. After they received superficial information, they did not understand or pursue it at a deeper level.

RETRACTED

#### 3.4.2. Criticism and Questioning

In response to bad information spread by new media, especially online social media, most students maintain an attitude of ignoring them and taking a casual look. A small number of college students will choose to respond directly to criticism or report to media monitoring platforms, such as WeChat, Weibo, and Zhihu media. That is, when most college students face bad information, they do not question or verify their behavior too much but maintain an irrelevant attitude, and their ability to criticize and question is particularly insufficient.

#### 3.4.3. Independent Thinking

When faced with information spread on various new media, about one-third of the students thought it was more credible, and at the same time, they would maintain their own ideas and do not blindly follow the trend. Some students remain skeptical about new media information and need to be verified, and only a small number of students fully accept the positive information that the public thinks. This shows that the surveyed students have a certain ability to think independently about the information disseminated by new media. A small number of college students never disseminate and forward unverified information. There are still many college students who spread unverified information on the Internet, and even some students directly forward and spread the information without further verification and confirmation of the source and authenticity of the new media information.

Independent thinking needs to be further cultivated and strengthened. About 10% of the students have participated in human flesh searches, spoofed pictures, dissemination of false or terrorist information, online verbal abuse or attacks on Weibo, Tieba, blogs, and other media. In the process of media participation, this part of college students has the phenomenon of unconstrained, unregulated, and weak moral and legal awareness. About 30% of college students are just casual and have no strong sense of participation. They are just simple media users and cannot use new media more actively.

Information fragmentation in the cross-media data analysis of college students based on DNN [24]. When users of new media participate in the production and dissemination of such information, they further diversify the dissemination subjects. When the focus of information dissemination shifts from the organizational level to the individual level, the main body of information production and dissemination also shows multidimensional growth, the entire information production is divided infinitely, and the information released in the absence of organized and specialized personal media and new media technology constraints. The information is fragmented. This information production mode leads to the complexity and crowding of the information environment while satisfying the changes of the audience's publishing rights and reading modes.

RETRACTED

### 3.5. The Elements of College Students' New Media Literacy

#### 3.5.1. Social Factors

The situation of college students is simple [25], and the social background is simple and closed. Therefore, when using new media, they often judge new media information based on their own experience. In the time of using new media, the average college students use mobile phones or computers to browse web information. In addition, to living in the school environment, students are more engaged in information activities in the new media environment created by new media, and this new media environment has a greater impact on their new media literacy.

#### 3.5.2. The Audience's Own Factors

The new media is not only the subversion of breakthroughs in electronic technology but also the changes brought about by it have triggered the transformation of social and life patterns in the society, and it is also an important force affecting the formation of contemporary college students' values. The Internet spirit [26, 27] represented by the new media, such as freedom, equality, and everyone's participation, is a universal value concept, which makes the college students awaken their awareness of rights and citizenship. In the new media era, the *individual interests* that were not valued in the past will have agglomeration effect and then form local *group interests*. Especially with the popularization of mobile Internet, news applications associated with Weibo, WeChat, and traditional media have gradually replaced the traditional one-way communication methods, and the sources of information are no longer limited to official releases due to their different communication methods. After the new media changes the traditional way of information dissemination, college students themselves can also be a media. Under the threshold of low cost and time-consuming training, they can have the power of the media to show themselves to a certain extent.

The age stage of college students makes their social experience, knowledge accumulation, and values in the formative period. However, with the reform and development of the social market economy, the wealth and interests of citizens are increasing day by day, and independent and diverse economic entities have begun to grow and become independent. Diversified interests have produced independent and pluralistic rights appeals. The wide application of new media enables college students to access more information and enables college students to participate in more opinions, and the emergence of college students follows. Diversity, decentralization, and self-esteem are characterized by values.

RETRACTED

### 3.6. Challenges in Cross-Media Retrieval

Cross-media retrieval technology [28, 29] has always been faced with many difficulties and challenges, and researchers have made many important contributions to this field by adhering to the spirit of perseverance in scientific research. As an important foundation of cross-media retrieval technology, DNN-based multimedia retrieval technology needs to process different types of multimedia data at the same time. These data are related in high-level semantics, but the underlying features have different structures [30, 31]. The heterogeneity of cross-media data [32] makes it impossible to directly calculate the relevance of different types of features, forming a semantic gap, which is also one of the urgent problems to be solved. This is the direction of future research, as shown in the figure below [33]. The challenges are content gap and semantic gap as shown in Figure 6.

## 4. Conclusion

With the growth of the Internet, college students naturally show a high media literacy towards new media. With the help of new media, college students use a variety of composite ways to express themselves and contact others, realizing convenient and efficient interpersonal communication. College students have expanded the established interpersonal relationships in real life to a variety of media. To master the characteristics of interpersonal communication of new media and make rational use of new media is a problem that cannot be ignored in the use of new media by college students. In the context of in-depth learning, the new media literacy analysis based on DNN has made important opportunities. This opportunity makes the public in the whole society must have higher requirements on media literacy, which also provides a better development field for media literacy education.

In future projects, we will verify number of cross-media retrieval technologies, extend them to the field of new media and to put forward new ideas for research. [34, 35].

## Figures and Tables

**Figure 1:** Cross-media topic text clustering for college students.

**Figure 2:** DNN structure.

**Figure 3:** The development trend of new media in China.

**Figure 4:** Three media commonly used by college students.

**Figure 5:** The weekly media time of college students.

**Figure 6:** Content gap and semantic gap.

**Algorithm 1:** Pseudocode of the optimization model.

**Table 1:** Course outline of MOOC's *new media literacy*.

Topics	Items	Class hour
1	Net-volution and its influence	2
2	Future journalism and future audiences	2
3	Internet public opinion: reality or illusion	4
4	How to avoid *stereotype*	2
5	Internet fake news	2
6	Sensationalism in the network	2
7	New media and consumer life	2
8	New media and citizen empowerment	2
9	New media and public advocator	1

RETRACTED

## Data Availability

The dataset used in this paper are available from the corresponding author upon request.

## References

[1] Campante F., Durante R., Tesei A. (2021). Media and social capital. *Annual Review of Economics*.

[2] Auxier B., Anderson M. (2021). Social media use in 2021. *Pew Research Center*.

[3] Zhu D., Chen S. New media communication of fashion consumer goods in the context of visual culture.

[4] Hu P., Fu R. (2022). Micro animation design based on new media app interaction. *Lecture Notes on Data Engineering and Communications Technologies International Conference on Cognitive based Information Processing and Applications (CIPA 2021)*.

[5] Oliver M. B. (2022). Social media use and eudaimonic well-being. *Current Opinion in Psychology*.

[6] Hameleers M. (2022). Separating truth from lies: comparing the effects of news media literacy interventions and fact-checkers in response to political misinformation in the US and Netherlands. *Information, Communication & Society*.

[7] Cannon M., Connolly S., Parry R. (2022). Media literacy, curriculum and the rights of the child. *Discourse: Studies in the Cultural Politics of Education*.

[8] Qiu L. (2015). *The world factory in the information age: the network society of the new working class*.

[9] Deng T., Hou X., Liu Y. (2021). Comprehensiveness, preciseness and interconnectedness: how to evaluate international public opinion based on cross-media data mining on the Internet. *Journal of Physics: Conference Series*.

[10] Li Y., Chen K., Liu S. (2022). Diversity and spatiotemporal dynamics of fungal communities in the rhizosphere soil of Lycium barbarum L.: a new insight into the mechanism of geoherb formation. *Archives of Microbiology*.

[11] Lu J., Plataniotis K. N., Venetsanopoulos A. N. (2016). Face recognition using LDA-based algorithms. *IEEE Transactions on Neural Networks*.

[12] Cai H., Yang Y., Li X., Huang Z. What are popular: exploring twitter features for event detection, tracking and visualization.

[13] Bian J., Yang Y., Zhang H., Chua T. S. (2015). Multimedia summarization for social events in microblog stream. *IEEE Transactions on Multimedia*.

[14] Wang Z., Li L., Zhang C., Huang Q Image-regulated graph topic model for cross-media topic detection.

[15] Jacobson L. P., Lau B., Catellier D., Parker C. B. (2018). An Environmental influences on Child Health Outcomes viewpoint of data analysis centers for collaborative study designs. *Current Opinion in Pediatrics*.

RETRACTED

[16] Lee E. E., Bangen K. J., Avanzino J. A. (2020). Outcomes of randomized clinical trials of interventions to enhance social, emotional, and spiritual components of wisdom. *JAMA Psychiatry*.

[17] Pumsirirat A., Yan L. (2018). Credit card fraud detection using deep learning based on auto-encoder and restricted Boltzmann machine[J]. *International Journal of Advanced Computer Science and Applications*.

[18] He Y., Xiang S., Kang C., Wang J., Pan C. (2016). Cross-modal retrieval via deep and bidirectional representation learning. *IEEE Transactions on Multimedia*.

[19] Latotzke C., Gemmeke T. (2021). Efficiency versus accuracy: a review of design techniques for DNN hardware accelerators. *IEEE Access*.

[20] (2022). China new media development report No.12. *Institute of Journalism and communication, Chinese Academy of Social Sciences*.

[21] Sanghera S., Neb T., Kaur S. P., Madan A., Singh B. (2021). Assessment and role of social media in dental education. *SPR*.

[22] Gupta R., Gupta P., Gupta S., Garg S. (2021). To evaluate the effect of Yoga intervention in reducing dental students’ anxiety prior to and during a periodontic surgical procedure. *Science Progress and Research*.

[23] Arshad A., Ghazal S., Saleem N., Hanan M. A., Arshad M. H. (2022). Revisiting media literacy measurement: development and validation of 3 factor media literacy scale. *Journal of Computer Assisted Learning*.

[24] Lee M., Ellis J. R., Keel C., Wickes R., Jackson J. (2022). When law-and-order politics fail: media fragmentation and protective factors that limit the politics of fear. *British Journal of Criminology*.

[25] Yilmaz M. B. (2017). The relation between academic procrastination of university students and their assignment and exam performances: the situation in distance and face-to-face learning environments. *Journal of Education and Training Studies*.

[26] Cavaliere F., Sircar R. P., Catuogno T. (2022). The future quantum Internet. *Quantum Computing Environments*.

[27] Majić T., Sauter M., Bermpohl F., Schmidt T. T. (2021). Connected to the spirit of the frog: an Internet-based survey on Kambô, the secretion of the Amazonian Giant Maki Frog (*Phyllomedusa bicolor*): motivations for use, settings and subjective experiences. *Journal of Psychopharmacology*.

[28] Jiang Y., Xue Z., Li A. (2022). Research on cross-media science and technology information data retrieval. https://arxiv.org/abs/2204.04887.

[29] Li A., Du J., Kou F. (2022). Scientific and technological information oriented semantics-adversarial and media-adversarial cross-media retrieval. https://arxiv.org/abs/2203.08615.

RETRACTED

[30] Huang Z. (2015). *Research on self-media recognition system based on support vector machine*.

[31] Sompoch P., XiaoYang C., Michiro K. (2001). Automatic recognition and location of road signs from terrestrial color imagery. *Proceedings of IEEE Geoinformatics & DMGIS*.

[32] Zhang C., Lei Y., Xiao X., Xinzhong C. (2022). Cross-media video event mining based on attention graph structure learning. *Neurocomputing*.

[33] Betke M., Makris N. C. Fast object recognition in noisy images using simulated annealing.

